RETRACTED

# Optimization Algorithm for Ideological and Political Curriculum Environment in Colleges Using Data Analysis and Neighborhood Search Operator

**DOI:** 10.1155/2022/5833589

**Published:** 2022-09-16

**Authors:** Chaoyuan Luo

**Affiliations:** ^1^School of Public Administration, South China University of Technology, Guangzhou 510640, Guangdong, China; ^2^School of Marxism, Guangzhou Huashang College, Guangzhou 511300, Guangdong, China

## Abstract

In the context of the new era, the distinctive function of BD (big data) analysis and prediction also introduces a new way of thinking to university IPE (ideological and political education), broadens the domain of university IPE, and enhances the curricular offerings of IPE universities. In order to enhance the intelligence and personalization of the intelligent teaching system, this paper describes in detail the design and implementation processes for each component of the system. It also uses the association mining rule algorithm of data mining. To maintain population diversity, a population initialization method and a neighborhood-based search operator are used, both of which are based on a thorough consideration of the characteristics of complex networks. The neighborhood search strategy enhances the local search capability of the TLBO (Teaching-Learning Based Optimization) algorithm. The optimized TLBO algorithm presented in this paper achieves the highest average modularity value of 0.5238 through testing on real-world data sets. The outcomes demonstrate that the algorithm performs well and is successful in identifying problems in the community.

## 1. Introduction

The growth of network information technology has allowed BD (big data) to permeate all spheres of life. Without a doubt, the inevitable rise of networked IPE is the era of BD (ideological and political education). BD is viewed as a value concept rather than a medium and a technical tool in the network IPE process [1]. It goes without saying that we must fully exploit the positive role of BD and achieve the organic integration of BD and IPE in order to improve the ideological and political theory course. Universities' IPE in the new era is also dealing with opportunities and difficulties brought on by BD. Currently, in IPE work in universities, the majority of the working hours are taken up by actual work. Through BD, individuals can examine BD sets devoid of random analysis, apply them to numerous societal fields, forecast and assess the direction of societal development, gain enormous value, and foster social advancement.

How to strengthen the deepening and integration of IPE in universities with the times has also become a new topic in the field of IPE. From the actual work of IPE educators, as the frontline workers of IPE work, their own IPE quality, theoretical level, and teaching methods are also uneven. The core feature of BD is its predictability. We can build data models based on information from various data sources, so as to predict the future development trend of things. Berry et al. pointed out that IPE workers should actively create a small environment in the social environment, which is of great significance to the development of educational objects and the smooth development of IPE activities [2]. Pan and Bi's exposition of the opportunities and challenges faced by universities' IPE in the era of BD is mainly manifested in the application of BD to lead universities' IPE to develop in a more scientific direction [3]. Zhang et al. mentioned the difficulties encountered in the integration of BD into universities' IPE, mainly the difficulties of shallow understanding, information screening, and talent shortage [4]. How should IPE workers explore the innovation and reform of the content system, methods, and extracurricular practice of IPE courses in universities in the new era? All these have become important practical issues that IPE discipline must pay close attention to and deeply study in the era of BD.

RETRACTED

What BD has is not a data fragment or a simple data accumulation, but a complete data set. The goal of realizing data-driven IPE is not only to solve the current problems, but also to innovate the IPE method system, explore new ways of IPE, and play a long-term role. It also enriches the connotation of university IPE system, makes contemporary university IPE work more scientific and more contemporary, and has important theoretical guiding significance for IPE practice research. The contributions of this paper are as follows: (1) This research is based on the network society in the new era, introduces the concept of data-driven as a comprehensive concept, and focuses on exploring university data-driven IPE, so as to enhance the strength and effectiveness of university IPE. (2) This topic is combined with the era of BD, and the research content has been innovated. The research explores the innovation of university IPE model in the era of BD from the perspective of the constituent elements of education model, closely follows the characteristics of the era of BD, takes solving practical problems as the starting point and the end result, and puts forward specific strategies for model innovation.

## 2. Related Work

### 2.1. Research on BD Technology

With the advent of the era of BD, the theoretical and practical research of BD is a hot and difficult point in various fields of society. Looking at the power of BD, the active implementation and design of national BD strategy, the wide application of enterprise BD, and the convenience brought to personal life are powerful driving forces for the development of BD. Through machine learning, the complementarity and integration of human beings and intelligent machines, artificial intelligence will help human beings transcend their own limitations, which is also the future of BD development.

RETRACTED

Shaobin et al. focused on the opportunity problem, thinking that we should study the essential characteristics of BD, innovate the research paradigm of network IPE, and combine macro coverage with micro deepening to cope with the arrival of BD era [5]. Jia and Dan think that the ideological and political orientation of BD are not very reliable, the data quality and results may be misleading, or the data cannot achieve the purpose of quantification [6]. Zheng believe that BD will replace the traditional carrier as a brand-new carrier of IPE, bringing about the second qualitative change of the carrier [7]. Wang and Zhang proposed and implemented an intelligent distance education platform environment based on multiple agents, which can realize the sub-adaptability and intelligence of a distance education system based on the web [8]. Wang analyzed the distribution of students' characteristics in the network environment and put forward the theoretical part of the user characteristics analysis system [9] by analyzing the static and dynamic information of learners in the learning process.

Lulat analyzed the practical application of BD IPE from the perspective of practice [10]. Clarke discussed the opportunities faced by university IPE in the era of BD from five aspects: relying on data to help improve the foresight, pertinence, scientificity, prevention, and orientation of IPE and discussed the challenges faced by university IPE in the era of BD from three aspects: talent shortage, backward technology, and personal information leakage [11]. Manzano suggested giving full play to the dominant position of classroom in university IPE, establishing the innovation mechanism of university IPE in the era of BD, and making scientific and rational use of data information and classroom [12].

### 2.2. TLBO Related Research

An algorithm for optimization called TLBO (Teaching-Learning Based Optimization) establishes the “teaching” process of teachers and the “learning” process between students. Many real-world issues have been successfully solved using its potent convergence and global search capabilities.

Zhang et al. introduced the reverse learning technology into the basic TLBO algorithm in view of the shortcomings of learners' learning process in TLBO, which not only improved the diversity of the population but also greatly reduced the possibility of the algorithm failing [13]. Hamzeh et al. regarded the ratio of the fitness value of iterative individual function to the fitness value of optimal individual function as a teaching factor and put forward an adaptive learning strategy. Reverse learning technology was introduced by Banu et al. to address the shortcomings of TLBO learners in the learning process [14]. This technology increased population diversity and successfully kept the algorithm from succumbing to local optimization [15].

RETRACTED

Sharma and Kumar used TLBO to solve continuous unconstrained and constrained optimization problems [16]. Bi and Pan put forward an optimal design scheme of plane steel frame by TLBO [17]. Ram et al. proposed an improved version of TLBO based on adaptive teaching factors and multiple teachers and applied the algorithm to multi-objective optimization of heat exchangers [18]. Shabanpour-Haghighi et al. used adaptive wavelet mutation strategy to update individual learners and used fuzzy method to update in external archive to control the size of archive when solving multi-objective power flow problem [19]. Hassanzadeh et al. combined PSO (particle swarm optimization) with GA (genetic algorithm) to solve the problems that PSO tends to fall into local optimum and premature convergence when solving combinatorial optimization, and they improved the local search ability of the algorithm by using crossover and mutation operations of GA [20].

## 3. Methodology

### 3.1. Analysis of the Challenges Faced by University IPE in the Era of BD

Education authorities and educational institutions at all levels have increased their focus on and investment in IPE, according to IPE managers. IPE managers now face opportunities and challenges in how to define the teaching objectives of educators and how to introduce and adapt teaching materials and methods according to different stages of social development. It is challenging to learn from practice and comprehend the essence and core of ideological and political theory due to the lack of social life practice. Or students may find themselves at a loss in the constantly shifting environment, unable to accurately capture their ideological trends and so on, because it is impossible to capture the corresponding technical means in time when the times are changing. Low labor productivity and an inadequate educational outcome are the results. In addition, students can easily access a variety of information in the era of BD, communicate with people more widely, and rely less on teachers.

College IPE classroom teaching is relatively simple and boring, and its educational content lacks novelty. It cannot fully absorb and utilize the information in various data sources, and it does not choose appropriate and effective BD for integration into daily teaching activities. Western capitalist countries will maintain growth for a long time. Although the economic growth of western countries slows down and their hard power declines, the competitiveness of soft power increases. Socialist core values will inevitably be affected, shaking the self-confidence and national pride that has been formed for a long time, resulting in the blind follow-up of western ideology and the confusion of its own values, and increasing the difficulty of IPE.

RETRACTED

BD has the characteristics of mass, speed, and diversity. In application, computer data processing ability is required, data compatibility processing is difficult, and optimization troubleshooting is unclear. This is the main dilemma of BD collection, storage, and solution. Most IPE disciplines are good at traditional words and deeds, but in the case of the Internet as a medium, there is a lack of opportunities for face-to-face communication, and many educational disciplines seem unable to do so. Today, many IPE staff often lack technical problems such as BD processing and analysis. Recognizing the importance of BD and improving information technology knowledge are the key for Internet IPE practitioners to overcoming their professional limitations.

Educational process is a dynamic process of information symbol transformation and dissemination in the two-way interaction between educators and educational objects. The arrival of the era of BD will inevitably lead to changes in the educational process. For example, in the era of BD, educational objects use the network to learn, and educators can extract and compare students' learning situations through fuzzy mining algorithms, explore the structure of defective behaviors, find factors and rules, and obtain information about students' learning effects. Whether and how the data can play the role of IPE need to be tested in practice. Data citation self-examination presents the activities of educators in this field online through charts and other means.

Information theory, also referred to as communication statistics theory, is a body of theories developed to address the issue of transmission process. The sender, the receiver, and the channel that connects them make up the information transmission system. The following uncertainty is this. It stands to reason that the ex post uncertainty is never greater than the ex post uncertainty and that it can never be lower. Information can only reflect the uncertainty of symbols, whereas information entropy, which is defined as follows, can be used to measure the overall uncertainty of the entire source X:

(1) $$\begin{array}{c} H\left(X\right)=P\left(a_{1}\right)I\left(a_{1}\right)+P\left(a_{2}\right)I\left(a_{2}\right)+\cdots +P\left(a_{r}\right)I\left(a_{r}\right)=-\sum P\left(a_{i}\right)|\log\;P\left(a_{i}\right). \end{array}$$

*r* is the number of all possible symbols of the source *X*; that is, the information entropy is defined by the average self-information provided by the source for each symbol.

RETRACTED

Let *X* correspond to the source symbol *a*_*i*_, *Y* correspond to the source symbol *b*_*j*_, and *p*(*a*_*i*_/*b*_*j*_) represent the probability that *X* is *a*_*i*_ when *Y* is *b*_*j*_.

(2) $$\begin{array}{c} H\left(\frac{X}{Y}\right)=-\sum_{i=1}^{r}\sum_{j=1}^{s}p\left(\frac{a_{i}}{b_{j}}\right)\log\;p\left(\frac{a_{i}}{b_{j}}\right)\text{.} \end{array}$$

Data mining (DM) is primarily used for evaluation, including evaluations of educational software, learning processes, teachers, students, and learning environments. The database is used to store different teaching resources, such as domain knowledge bases, student information bases in student models, cognitive state bases, and learning history bases.  Figure 1 depicts the model of an intelligent teaching system based on the web.

Among them, DM module is the key component of building an intelligent distance learning environment, which mainly analyzes the data in the student information base and provides the discovered patterns and rules for the knowledge base. This module is mainly composed of four parts: preprocessing module, algorithm module, display module, and feedback module.

A statistical classification technique called Bayesian classification can forecast the likelihood that a given sample will fall into a particular category. Its performance is on par with that of neural networks and decision trees in some fields. The Bayesian theorem serves as the foundation for Bayesian classification.

Assuming that there are *m* classes {*C*_1_, *C*_2_, ⋯, *C*_*m*_}, then the condition of assigning sample *X* to class *C*_*j*_(1 ≤ *i* ≤ *m*) is *P*(*C*_*i*_*|X*) > *P*(*C*_*j*_*|X*), *j* = 1,2, ⋯, *m*, *j* ≠ *i*. That is, the probability that the sample is assumed to be class *C*_*i*_ is greater than that of other classes. According to Bayes theorem,

(3) $$\begin{array}{c} P\left(C_{i}|X\right)=\frac{P\left(X|C_{i}\right)P\left(C_{i}\right)}{P\left(X\right)}\text{,} \end{array}$$

where *P*(*X*) refers to the probability that any data object conforms to sample *X*, which is constant for all classes.

Given the sample's class label, it is presumed that the attribute values are conditionally independent of one another or that there is no dependency between the attributes, allowing the calculation of *P*(*X|C*_*i*_) to be performed using the following formula:

(4) $$\begin{array}{c} P\left(X|C_{i}\right)=\prod_{k=1}^{n}P\left(x_{k}|C_{i}\right)\text{.} \end{array}$$

The results show that Bayesian classifier has a good classification effect on two kinds of data: one is completely independent data, and the other is functionally dependent data.

RETRACTED

### 3.2. University IPE Path Optimization

IPE is currently taught primarily through classroom indoctrination, and student evaluations are primarily based on test scores. Teachers must reconsider their initial assumptions because in the era of BD, this method can no longer satisfy IPE requirements.

The rise of data-driven concept has broken people's traditional thinking. And thoughts and behaviors can be presented in the form of intuitive and quantitative data. University IPE has given way to great innovation and development. Therefore, the subjects and objects of university IPE should change their thinking in time, establish the idea of data-driving, break through the limitation of time and space, improve the ability of data analysis and application, and focus on individualized education. Educators must realize the expansibility of data-driven educational space, which makes it multidimensional and open. Education space is the place where both sides of education carry out educational activities. Data-driven educational space is moving from “closed” to “multidimensional” and “open.” Supported by powerful data screening and analysis functions, it can accurately analyze students' ideological and behavioral trends, timely feed back data, and provide technical support for ideological and political work. Furthermore, ideological and political workers in universities are encouraged to use data technology to apply, improve, and test data ability in practice, so as to improve the times and initiative of ideological and political work.

In the era of BD, network IPE workers need not only a high level of political theory, but also the ability to deal with the rapid spread of information, which requires educators to effectively master network technology and network cultural characteristics. Providing diverse and comprehensive services through data processing platform and perfect front-end service platform will greatly improve the actual work efficiency of educational subjects with heavy daily workload. From the perspective of BD application, the key is to establish and improve the working mechanism of interaction and coordinated development among managers, educators, and students. This way, a teaching resonance is formed with college students and truly realizes the IPE of thoughts and hearts. At the same time, by using the insights generated by college students' behavior data, we can also optimize the management ways and methods of student administrators in students' daily management.

RETRACTED

In both daily life and work, decisions must frequently be made. The classic single-objective optimization problem arises when people use decision rules (objective functions) to make a given decision “optimal” in the sense of the decision rules. Finding a decision variable vector and optimizing the vector made up of objective functions while taking into account all constraints are how the multi-objective optimization problem is usually defined. Generally speaking, the multi-objective optimization problem can be described by the following mathematical model, using minimization as an example:

(5) $$\begin{array}{c} Min\left\{f\left(x\right)\right\}=\left[f_{1}\left(x\right),f_{2}\left(x\right),\cdots ,f_{M}\left(x\right)x\in D\right]\text{,} \end{array}$$

where *f*(*x*)=[*f*_1_(*x*), *f*_2_(*x*), ⋯, *f*_*M*_(*x*)] is the objective vector, *f*_*i*_(*x*)(*i*=1,2, ⋯, *M*) is the *i*th objective function value, and *Min* is the minimization of the objective vector.

For a given multi-objective optimization problem, let its domain be *D*; then, the Pareto optimal solution set *x*^*∗*^ ∈ *D* is as follows:

(6) $$\begin{array}{c} x^{*}=\left\{x\in D|\neg \exists x^{\prime }\in D,f\left(x^{\prime }\right)<f\left(x\right)\right\}\text{.} \end{array}$$

A multi-objective optimization problem must have a Pareto optimal solution in order to have an optimal solution. The TLBO algorithm first generates a set of initial student score values at random for the search space. Students assist and learn from one another as they study, which helps to improve one another's performance to some extent. After the two processes mentioned above, students' achievement can be significantly raised and can even approach that of teachers. The first process relies heavily on the difference between teachers' and students' average grades to raise students' grades. Namely,

(7) $$\begin{array}{c} {\text{Different\_mean}}_{i}=r_{i}\left(X_{teacher}-T_{F}\cdot M_{i}\right)\text{,} \end{array}$$

where *r*_*i*_ is a random number in the range of [0, 1] and teaching factor *T*_*F*_ = *round*[1 + *round*(0,1){2 ~ 1}], that is, a random value between 1 and 2.

Select two students *X*_*i*_, *X*_*j*_ at random. When *X*_*i*_'s grade (*X*_*i*_′) after the teaching process is better than *X*_*j*_'s grade (*X*_*j*_′) after the teaching process, update the current grade to *X*_*new*_ with the following formula:

(8) $$\begin{array}{c} X_{new}=X_{old}+r_{i}\left(X_{i}-X_{j}\right)\text{.} \end{array}$$

The final score must be established by comparing the fitness values rather than accepting the updated score as the final score. And when the fitness value of *X*_*new*_ is better than *X*_*old*_, the *X*_*old*_ is updated; otherwise, the original value is kept.

RETRACTED

If the target learners are long-term users, they can analyze the courses they are interested in according to some basic information, such as study records and professional codes, and then make suggestions. Compare the information with different groups of learners. According to the principle of maximum similarity, find the group with the same preference as the target learners, and then recommend the next step. The entities contained in the student achievement management information system mainly include departments, teachers, classes, students, and courses. The relationship between them is described by ER diagram, as shown in Figure 2.

The application of DM in students' course performance analysis mainly analyzes the shortcomings of existing course performance analysis and applies association rule mining technology to students' performance analysis, aiming at determining the relationship between course setting and course performance on the platform network and discovering the important information hidden between the networks. Therefore, the change of IPE thinking in the era of BD mainly aims at the general changes of students and makes some specific adjustments to individual education.

The basic TLBO algorithm shows good performance in solving simple low-dimensional problems, with fast solving speed, high precision, and good global searchability. However, when solving relatively complex multimodal problems, the global searchability is poor, and it is likely to fall into local optimization. In view of these shortcomings of TLBO algorithm, this paper proposes a TLBO with self-learning ability. This algorithm refers to the main idea of harmony search algorithm and introduces the concept of “self-learning” of students to improve, thus improving the overall searching ability of the group.

In this paper, *mean* is improved to make *mean*=*x*_*worst*_+*x*_*i*_/2, which makes the value of *mean* different for individual *X*_*i*_ in the teaching process, thus ensuring the diversity of population and preventing premature convergence of the algorithm, as follows:

(9) $$\begin{array}{c} T_{F_{i}}=\text{round}\left[1+\text{round}\left(0,1\right)\right]\text{,}\\ {\text{Different\_mean}}_{i}=r_{i}\left(X_{teacher}-T_{F_{i}}\cdot \text{mean}=\frac{x_{worst}+x_{i}}{2},i=1,2,\cdots ,\text{NP}\right). \end{array}$$

Everyone learns in the best way through self-adjustment. As each student can take several courses at the same time (multi-decision variables), only some subjects will be adjusted and studied during “self-study,” while the dominant subjects will be retained and the inferior subjects will be promoted. The flowchart of the algorithm is shown in Figure 3.

RETRACTED

The specific steps are as follows:

1. Initialize the population number.
2. Calculate the fitness value and average score of each student, and determine the teacher.
3. Judge whether to accept the teaching result by the fitness function before and after teaching.
4. Learning process: Students with the fitness value of the top 5% are selected and set as top students. Students who skip the teaching process will communicate with these students to improve their grades.
5. Execution process validity judgment: if it is less than the maximum iteration number, return to step 2; otherwise, output the optimal solution.

## 4. Experiment and Results

This work replicates two common real-world restricted optimization problems to test the performance of the proposed TLBO algorithm. The experiment's final criterion for an algorithm is its maximum number of iterations, and all algorithms have a maximum of 100 iterations. The top solutions sought by various algorithms are displayed in Table 1.

It can be seen that if the corresponding volume is required to be the smallest, GA will find the minimum value of 0.0044 m^3^, while the optimized TLBO will find the value of 0.0041 m^3^. If the corresponding pressure is required to be the minimum, the stress sought by the optimized TLBO is the minimum, which is 8427.36 kPa. Therefore, the optimized TLBO algorithm has achieved a good optimization effect on the stress value.

Figure 4 shows the statistical mean values of the solutions obtained when 24 10-dimensional benchmark functions are independently run by different optimization algorithms 60 times. Compared with other algorithms, the optimization performance of optimized TLBO is superior to that of *w* functions.

The comparison results show that TLBO optimization can achieve the ideal optimal solutions of reference functions 7, 8, 9, 16, and 17. The proposed optimized TLBO significantly improves the computational performance of TLBO, although the optimized TLBO is not always superior to other algorithms. The traditional learning algorithm cannot meet the requirements of recognition accuracy and convergence speed of the system. With the rapid development and wide application of intelligent computing methods, people actively seek to use intelligent computing methods to determine the model structure and model parameters of nonlinear systems, so as to improve the system identification performance.

RETRACTED

For four real-world data sets, the TLBO algorithm and the single-objective optimization technique are contrasted in this section. The experimental findings for modularity mean are displayed in Figure 5.

For Dolphins network, the TLBO algorithm proposed in this work has the highest average modularity value of 0.5238, which shows that in Dolphins network, the optimization result of TLBO algorithm is the best, and the network community structure is stronger. The average values of GA, PSO, and Bayesian algorithms are 0.4003, 0.3122, and 0.3122, respectively, and the optimization results are obviously inferior to those of TLBO algorithm. In the TLBO algorithm proposed in this paper, considering the characteristics of community network, the population initialization method and neighborhood search method are adopted to keep the diversity of the population.

When a node has no power, its neighbors will wake up, so the detection coverage and the number of active nodes will be monitored simultaneously. The same network sample nodes and unified target point deployment are used for simulation, and the performance of TLBO algorithm is compared with the other three algorithms.  Figure 6 shows the inspection coverage and the number of rounds.

It clearly shows that GA and PSO algorithms cannot keep the detection coverage. At 300 rounds, the TLBO algorithm can maintain 100% coverage. Between 400 and 900 rounds, the results of TLBO and Bayes are similar, but the Bayesian algorithm has 70.1% coverage at 900 rounds. The advantages of TLBO algorithm increased significantly from 1000 rounds, while the network life was extended to 1600 rounds. The modeling errors of the four methods obtained are shown in Table 2.  Figure 7 shows the error comparison of the modeling results of the four modeling methods.

It can be seen that the model established by the optimized TLBO is more consistent with the real value. This further illustrates the effectiveness of the algorithm proposed in this paper in modeling application. The modeling method in this paper is data-driven, easy to implement, and also applicable to the modeling of other chemical processes.

The comparison results in Figure 8 show that for a 30-dimensional optimization problem, all optimization algorithms have the same optimization results for reference functions 7 and 9 and all optimization algorithms have found an optimal solution. Test the global ideal of function 9.

It can also be seen that compared with TLBO, all other hybrid optimization algorithms have better, or at least equivalent, solution accuracy for single-mode optimization problems and some complex multimode optimization problems. The accuracy of other optimization algorithms is better than that of TLBO. For the reference function 9, all algorithms converge to the global optimal solution.

RETRACTED

Information resources can only play a role through carriers, and related technologies can only realize their own value by carrying information. Therefore, how to promote the integration of information resources and technical resources is crucial for IPE resource allocation in the era of BD. To make rational use of IPE's BD resources, the related resource management system is the necessary support for its existence. The computerization and digitalization of IPE resource development mainly include the networking and intelligence of resource development. Infrastructure construction is the basic guarantee for the informatization of eco-industrial park resource development. To realize the combination of online and offline IPE resource allocation, make the school IPE allocation flexible and dynamic.

Higher standards for college students are introduced by the application of BD in university EPI, in addition to additional obligations for educational administrators and educators. College students have access to a variety of knowledge sources in the BD era. Students now receive their education from more sources than just teachers and textbooks. The autonomous learning mode is a crucial way to boost universities' subjective initiative. However, offline educators must also provide oversight for online learning. In the era of BD, the combination of the two can significantly enhance college students' learning outcomes.

## 5. Conclusions

In the era of BD, IPE process and data insight are the sources of all value. The dawn of the BD age has had a significant impact on every field in the globe, and the fusion of BD and education will result in significant shifts in the educational landscape. We can fully utilize the information and optimize the relationship between knowledge points by integrating artificial intelligence, distributed learning, and network technology into the system. This is done by taking into account each student's unique cognitive abilities, knowledge point errors, learning needs, and interests. As a result, this work designs appropriate discretization algorithms for various issues and suggests appropriate discrete TLBO. The simulation results demonstrate that in the Dolphins network, the TLBO algorithm has the best optimization impact and the strongest network community structure, as it can achieve the greatest modulus average of 0.5238 using the optimal TLBO approach suggested in this study. Alter one's way of thinking, continually enrich the curriculum, reinvent the delivery method, enhance the instructional techniques, and pay close attention to the ongoing practice and administrative procedures of ideological work in universities.

RETRACTED

## Figures and Tables

**Figure 1:** Web-based intelligent teaching system model.

**Figure 2:** ER diagram.

**Figure 3:** Flowchart of optimizing TLBO algorithm.

**Figure 4:** Comparison of test function optimization results.

**Figure 5:** Modularity value obtained in real network.

**Figure 6:** Relationship diagram between node coverage and node life cycle.

**Figure 7:** Error comparison of modeling results.

**Figure 8:** Comparison of optimization results of different mutation strategies.

**Table 1:** Simulation test results of different algorithms.

Algorithm	min(*f*_1_)	max(*f*_2_)	max(*f*_1_)	min(*f*_2_)
Optimized TLBO algorithm	0.0041	9632.21	0.0568	8427.36
GA	0.0044	9963.25	0.0537	8432.14
PSO	0.0046	9863.39	0.5029	8469.74
Bayesian classifier	0.0049	9698.27	0.0527	8455.19

**Table 2:** Modeling error of multiple algorithms.

Algorithm	Error interval	MSE
Optimized TLBO algorithm	[−0.0563,0.0041]	0.0063
GA	[−0.0768,0.0056]	0.0096
PSO	[−0.0821,0.00501]	0.0241
Bayesian classifier	[−0.0968,0.00528]	0.0368

## Data Availability

The data used to support the findings of this study are available from the author upon request.
